The article "Application of Decision Tree Intelligent Algorithm in Data Analysis of Physical Health Test" was published in 2022. Journal: J Healthc Eng.

# Application of Decision Tree Intelligent Algorithm in Data Analysis of Physical Health Test

**DOI:** 10.1155/2022/8584377

**Published:** 2022-01-11

**Authors:** Li Chen, Meiling Miao

**Affiliations:** ^1^School of Physical Education and Health Science, Chongqing Normal University, 401331 Chongqing, China; ^2^Sichuan University, Chengdu, China

## Abstract

With the continuous development of China's cultural industry, people's health has become one of the topics of the highest concern. Therefore, all the application models of physical health test data in the actual analysis have become the current research focus and trend direction of healthy constitution. This paper summarizes the significant problems in the analysis of physical health test data, through the comprehensive analysis and investigation of physical health test data, combined with the measurement of the test indicators, through the analysis and processing system of youth physical health data, the use process of national youth group physical health standard data management software, and decision tree intelligent algorithm in physical health. The research steps of test data analysis and application model summarize the application characteristics of physical health test data in the application process. Based on this, a decision tree intelligent algorithm is proposed, and the corresponding functions and optimization formulas of the algorithm are substituted. In the process of actual sample checking calculation, each weight range and corresponding errors are inferred and analyzed by combining examples. This paper summarizes the application model and optimization model of health test data analysis based on decision tree intelligent algorithm. Through the repeated test of the research data, the feasible area and application scope of the algorithm are obtained, and the practical optimization scheme and application ideas under the algorithm are obtained.

## 1. Introduction

With the continuous expansion of our country's control over physical health, our achievements in physical health testing have gradually become the focus of attention of all sports groups and show an excellent development trend. However, in the application process of the data analysis of the physical health test, there are often some abnormal problems such as the athlete's physical health test mode and incomplete data analysis, which are obviously reflected in the data analysis process of the physical health test. Therefore, in the questionnaire survey, we can use association rules to explore the rules in the actual physical health test process and take this as the analysis data to calculate the actual evaluation index and its health rules under the quantitative table and draw the conclusion that each worker in the questionnaire has two or more positive psychological problems, mainly manifested as depression and obsessive-compulsive disorder. According to the particularity of the symptom, an effective scheme under the association rule algorithm is inferred [1].

This paper focuses on the current detection modes of physical health test, discusses how to reflect the difference of physical health test data and its physical condition comprehensively, analyzes the decision tree intelligent algorithm and the application model of physical health test data analysis under the algorithm in combination with various vector and variable indexes, and finally summarizes the optimal model of physical health test data. On this basis, the algorithm function of each research index is substituted to carry out the survey of each test area, and the element indexes under the behavior detection algorithm are integrated and classified. After repeated verification, combined with relevant parameters, the key measurement steps in the research are applied to get the actual optimized operation mode under the benefit.

The innovative contribution of this paper is that, based on the development status of health testing, an innovative decision tree intelligent algorithm and its optimized application function are proposed, which is substituted into the analysis process of physical health testing. Through data analysis, the application distribution range and actual operation mode of each physical health test data are obtained, and the basic upgrade indicators under this test are summarized. Based on the algorithm, various optimization modes are investigated on the spot, and the benefit analysis is carried out according to the actual situation. By introducing various parameter data and experimental results, the application model of decision tree intelligent algorithm in physical health test data analysis is summarized.

The structure of the article is divided into three parts. Among them, the second part focuses on the comprehensive discussion of the decision tree intelligent algorithm mode based on the analysis of the physical health test data, including the decision tree intelligent algorithm and the physical health test data analysis system; the third part carries out the field investigation and questionnaire survey on the established decision tree intelligent algorithm model and calculates the specific analysis of the physical health test data under the algorithm. The application form, through continuous checking and comprehensive analysis, summarizes the corresponding experimental data and research results, so as to prove the optimal research model under the algorithm and finally collects all the effective experimental data integration to build the optimal application model of decision tree intelligent algorithm in the analysis of physical health test data.

## 2. Related Work

In recent years, many scholars and researchers have carried out detailed research on decision tree intelligent algorithm and physical health test data analysis system and obtained the corresponding research results after substituting each index and step into the research data. Li et al. analyzed the actual classification and attribute characteristics under the form according to the employment mode of each college student, determined the data processing rules and employment form characteristics under the attribute, combined with the actual mining technology of preprocessing and information data, and summed up the intelligent algorithm model and optimization form of the decision tree under the simple structure [2]. By analyzing the actual behavior and performance of students in the process of movement, it was proposed to substitute the algorithm advantages of decision tree into each motion structure and obtain the optimal motion analysis form under the decision tree algorithm model [3]. Zhang et al. introduced various algorithms to the actual network model of various medical images, combined with PCNN parameters to carry out information processing on segmentation processing and visual resolution of fitness test, and summarized the high-precision processing parameters under the scientific and technological conditions of the algorithm [4]. Guo et al. conducted concept differentiation and subset classification on the attributes and data characteristics of the research objects and analyzed the medical data management system based on physical health with various management statistical methods to further improve the data management efficiency and basic level [5]. Kumar and Senthil expressed the needs for the evaluation of students' emotional quality, differentiated the learning samples and data records, substituted the category nodes mapped by the model in the decision tree algorithm, and completed the actual supervision of emotional quality under the algorithm with this branch [6]. After searching the knowledge base of data mining, Yahaya et al. proposed optimizing the decision tree algorithm, Bayesian classification, and support vector machine and then applied them to the actual measurement process in various fields, so as to predict the health status of the research object [7]. Wang et al. focused on the research field of medical data analysis, tested the data analysis tools and application technologies in the database, summed up the problems and causes in the process of analysis of physical health data, and concluded the typical advantages of this analysis method [8].

Baldwin et al. proposed the application of ID3 learning algorithm of probability fuzzy decision tree based on quality allocation in practical functions. In the algorithm, the actual application of the quality and complexity evaluation of theoretical association is combined with examples, and the discrete characteristics of the algorithm are verified [9]. Liu et al. applied the intelligent evaluation algorithm to the anesthesia depth detection system and obtained the actual parameter changes of each patient during the anesthesia period from the physical health test gap after the combination of the system, so as to verify the feasibility of the algorithm [10]. PAAP et al. comprehensively tested the performance of computer adaptive testing, so as to carry out model analysis and data integration for multidimensional projects. Through the evaluation of the patient database in the field, the optimal response use model at this level was obtained [11]. Combining the health risks of Mexican women in the postpartum period, Jewel et al. conducted a general survey on more chronic health diseases and found that there are specific differences in age, language, and family income among women in different income families, which are used as interactive data support to verify the health maintenance rules that can increase each output index [12]. Combined with the actual development of economy, politics, technology, society, and other fields, Russo et al. conducted a comprehensive investigation on the occupational physical and mental health and occupational risks of employers and summarized the actual linear regression analysis scheme under this sample [13]. Allen MS and others proposed that individual physical activity has an important impact on the quality of life. Through the establishment of the potential score table of physical activity and the two-way table of personality self-evaluation, the related impact of physical training on physical health was tested in an open way, and the corresponding test results were obtained [14]. Nurius et al., based on a hypothetical framework of stress theory, tested and investigated various risk factors, showed the characteristics of the population under the equation structure by various structure fitting tests, and summarized the maintenance role of stress process in actual physical health [15]. However, the above research introduces the characteristics of decision tree intelligent algorithm and physical health test data analysis system from different perspectives but lacks the actual analysis process and results under other algorithms, and the research on its application scope is not comprehensive. Therefore, based on the existing effective research data, this paper comprehensively studies the solution of physical health test number under the decision tree intelligent algorithm from the perspective of algorithm, according to the existing problems in the actual program, to improve the establishment of decision tree intelligent algorithm under the optimal calculation model.

## 3. Application Model of Decision Tree Intelligent Algorithm in Physical Health Test Data Analysis

### 3.1. Analysis and Application of Physical Health Test Data

The physical health test data is the basic information stored in the national standard data management database, and in the actual measurement, it shows the specific decomposition of each body type, health status, and disease characteristics, so as to show the index under the characteristic test and its checking calculation results. Therefore, after analyzing the comprehensive indicators of the physical health test data in China, it is not difficult to find that the analysis of adolescent physical health test data, as the most important part of the application model research of physical health test data analysis, has a certain level and status in the actual basis. Therefore, when analyzing the application scope of the group's physical health test data, first of all, it is necessary to conduct comprehensive statistics on the group's physical health test indicators, so as to obtain the basic indicators of physical health, as shown in Table 1.

From Table 1, the analysis and application of physical health test data are mainly reflected in the analysis and processing system of adolescent physical health data, and the specific performance in the indicators is the system category. The system category includes user management, data upload, data processing, and data standard management. Among them, the specific indicators of user management are user account management and user information management; the specific indicators of data upload are body test score entry and body test score import; the specific indicators of data processing are body test data increase, body test data deletion, body test data modification, and body test data query; the specific indicators of data standard management are body test index management and scoring standard administration. From the above indicators, we can get the following procedures for the use of data management software for national youth group physical health standards, as shown in Figure 1.

Figure 1 shows the use process of data management software for national youth group physical health standards, which shows the process from input to output. First, import the data, submit the verification file, input and save the basic information, then get the data registration card by setting the test item, filling in the serial number of the instrument, inputting the test result, modifying the format file, reviewing the test result, calculating the evaluation score, and generate the report file by data export and backup, so as to connect the network to upload the final data. Among them, the input of test results into the corresponding format file contains the data results generated by the system and other software, which are divided into manual input, test instrument input, and palmtop computer input. Therefore, the use process as a basic index of physical health calculation means, in the actual use process, has excellent applicability.

### 3.2. Intelligent Algorithm Model of Decision Tree

In the basic index of physical health and the use process, the intelligent algorithm model of decision tree is substituted to get the characteristic attributes of the index and the potential laws of the data. Taking the generated samples of decision tree as the judgment boundary point, the optimal threshold of each accuracy is calculated, and the high-precision decision tree analysis mode is obtained. The basic information model of decision tree is obtained by the data sorting function of each node. Therefore, the training sample set of the information model is regarded as a whole, with *m* as the number and *C*_*i*_ as the category. Among them, *i*=1,2,…, *m*, the expected information function in the set *S* is

(1) $$\begin{array}{c} I\left(r_{1},r_{2},\ldots ,r_{m}\right)=-\sum_{i=1}^{m}p_{i}\log_{2}\left(p_{i}\right). \end{array}$$

In the above formula, *R*_*i*_ represents a subset of *C*_*i*_ categories in data set *S*, the number *C*_*i*_ of them is represented by *r*_*i*_, and *p*_*i*_ represents the probability of belonging to *C*_*i*_ category after random sample extraction, which conforms to *p*_*i*_=*r*_*i*_ ÷ |*S*| rule. If the attribute *v* is divided into two different subsets of data, and there are classification rules of *i*=1,2,…, *v*, then the attribute value *a*_*j*_ in the *A* attribute can be divided into different branches and expressed in the *m* category group as follows:

(2) $$\begin{array}{c} E\left(A\right)\sum_{j=1}^{v}\frac{S_{1j}+\cdots +S_{mj}}{\left|S\right|}I\left(S_{1j}+\cdots +S_{mj}\right), \end{array}$$

in which

(3) $$\begin{array}{c} W_{j}=\frac{S_{1j}+\cdots +S_{mj}}{\left|S\right|}, \end{array}$$

where *W*_*j*_ is the specific gravity value in the subset *S*_*j*_. Then, this subset class *C*_*i*_ is substituted into the expected information function, and the calculation formula is as follows:

(4) $$\begin{array}{c} I\left(S_{1j}+\cdots +S_{mj}\right)=-\sum_{i=1}^{m}p_{1j}\log_{2}\left(p_{1j}\right), \end{array}$$

in which

(5) $$\begin{array}{c} p_{ij}=\frac{S_{ij}}{S_{j}}. \end{array}$$

In the above formula, *I*(*S*_1*j*_+⋯+*S*_*mj*_) represents the expected information amount of *C*_*i*_ category in *A* attribute and *S*_*ij*_/*S*_*j*_ represents the proportion value of *S*_*j*_ subset in *S*_*j*_ category. Therefore, through the above function formula, taking attribute *A* as a whole, the information gain measure function in the decision classification attribute is calculated as follows:

(6) $$\begin{array}{c} \text{Gain}\left(A\right)=I\left(r_{1},r_{2},\ldots ,r_{m}\right)-E\left(A\right). \end{array}$$

In the above formula, after the whole data set is divided into different subsets, the deviation on variables is particularly obvious. Therefore, after substituting the deviation index, the optimized function is calculated as follows:

(7) $$\begin{array}{c} \text{SplitInfo}\left(S,v\right)=-\sum_{i=1}^{m}\frac{\left|S_{i}\right|}{\left|S\right|}\times \;\log_{2}\frac{\left|S_{i}\right|}{\left|S\right|}. \end{array}$$

From the above formula, we can deduce the optimized information gain rate function, that is, the maximum information gain rate function, which aims to complete the determination of the criteria for the partition of sample attributes and make up for the deficiencies and so on, which is expressed as follows:

(8) $$\begin{array}{c} \text{GrainRatio}=\frac{\text{Grain}\left(s,v\right)}{\text{SplitInfo}\left(s,v\right)}. \end{array}$$

On the basis of samples, combined with each prediction index, the function value fields under different categories are calculated, where for *C*(*i*), as the sample miscalculation cost, the function formula of its category is

(9) $$\begin{array}{c} C\left(i\right)=\sum_{j,i=1}^{m}\cos\;t\left(i,j\right). \end{array}$$

In the above formula, cos  *t*(*i*, *j*) is *i*=*j*/*i* ≠ *j*. *w*(*i*) is used as the weight value in the *u*_*i*_ sample category. The function formula of the category is

(10) $$\begin{array}{c} w\left(i\right)=C\left(i\right)\frac{n}{\sum_{k=1}^{m}C\left(k\right)n_{k}}. \end{array}$$

In the above formula, *m* is the number of values, *n* is the total number of samples, and ∑_*k*=1_^*m*^*C*(*k*)*n*_*k*_ is the sum of the maximum category weight values under the decision tree model if it is equal to *n*. The maximum benefit function of *p*_*i*_ probability is obtained as follows:

(11) $$\begin{array}{c} \left\{\begin{array}{c} p_{i}=\frac{W_{i}}{\sum_{i=1}^{m}W_{i}}=\frac{w\left(i\right)n_{i}}{\sum_{i=1}^{m}w\left(i\right)n_{i}}\\ p_{ij}=\frac{w\left(i\right)n_{ij}}{\sum_{i=1}^{m}w\left(i\right)n_{ij}} \end{array}\right.. \end{array}$$

Therefore, by setting each index coefficient, the index calculation function of the expected information and the category weight value in the above decision tree algorithm model calculates the corresponding optimal index function after substituting the category difference and error index and presents the optimization trend in each index cost weight value field, effectively reducing the probability of error generation, and improving the decision tree in each. The application value field of the system is time-effective.

## 4. Experimental Design and Analysis

Based on the current situation of the development of the analysis and processing system of the physical health data of various groups in China, this paper makes a comprehensive analysis and on-the-spot investigation on the adolescent groups. Through the calculation of the physical health evaluation model, which is mainly based on the factors of body mass index score, vital capacity single score, and gender difference characteristics, it distinguishes between the actual results and the specific research data. In order to get more and more accurate results of research data, we can build a practical project model with the least error and the highest benefit. In this study, the students from freshmen to seniors of a university in China are taken as the research objects. Firstly, the statistical analysis data of the calculation samples of each grade of the university are calculated, as shown in Figure 2.

Figure 2 shows the analysis and distribution diagram of the decision tree intelligent algorithm model introduced into the student group in the study school area, in which the research object is divided into two research perspectives, male and female, according to the gender standard. The total number of samples studied on the campus is considered as a whole, which is 100%. The experimental steps are divided into two groups: tested and non-tested. The weight of tested boys is the largest in the total sample number, followed by tested girls, test-free boys, and test-free girls. Its form shows that the proportion of the total number of samples in the research data of the campus is very large in the actual research and analysis process, which can show the integrity in the data, and through this statistical data, the actual distribution proportion of tested boys and tested girls is obtained, as shown in Figure 3.

Figure 3 shows the proportion of male and female in adolescent physical health test data analysis after substituting decision tree intelligent algorithm. It is centered around the center of the circle and spreads around, showing a value of 0–90 around the circle. Among them, the first circle is a freshman, the second circle is a sophomore, the third circle is a junior, the fourth circle is a senior, and the values are constantly changing within 0–90. And the connecting line from the center of the circle to the surrounding area shall prevail. The left area in the figure shows the proportion of female students, and the right area in the figure shows the proportion of male students. It can be seen from this that the numerical range of boys is lower than that of girls, and there is an unbalanced distribution. Combined with the reality, it may be that boys have the habit of smoking and drinking, which leads to the poor physical health data compared with girls. On this basis, the body mass index of each grade is also included in the study, and its score is used to analyze the physical health of the study object. The data are as follows.

Table 2 shows the test data of adolescent body mass index after the intelligent algorithm of decision tree, in which freshmen to seniors are taken as the research category; the low weight range of freshmen is ≤13.4, the low weight score is 80, the normal range is 13.5–18.1, the normal score is 100, the overweight range is 18.2–20.3, the overweight score is 80, the obesity range is ≥20.4, and the obesity score is 60; the low weight range of sophomores is ≤13.6, the low body weight score is 80, the normal range is 13.7–18.4, the normal score is 100, the overweight range is 18.5–20.4, the overweight score is 80, the obesity range is ≥20.5, and the obesity score is 60; the low body weight range of juniors is ≤17.8, the low body weight score is 80, the normal range is 17.9–23.9, the normal score is 100, the overweight range is 24–27.9, and the overweight score is 80, The range of obesity is ≥28, and the score of obesity is 60; the low weight range of seniors is ≤17.1, the score of low weight is 80, the range of normal is 17.2–23.9, the range of normal is 100, the range of overweight is 24–27.9, the range of overweight is 80, the range of obesity is ≥28, and the score of obesity is 60. Therefore, the value of low weight range is the highest among junior boys, the value of normal range is the highest among junior boys, the value of overweight range is the highest among junior boys and senior girls, and the value of obesity range is the highest among junior boys and senior girls. Similarly, in other physical health test data such as vital capacity, the value of freshmen and sophomores is lower, and the value of freshmen, sophomores, and seniors is also the highest. At the same time, the value in the table is basically the same as that in the obesity range.

Therefore, by analyzing the obesity value, gender difference, and other physical health test data that affect the physical health test data, it is found that once the scores of each index are used to repeatedly verify the youth physical health test data under all the decision tree intelligent algorithms, the decision tree intelligent optimal algorithm and its application mainly focus on the research of the application model of physical health test data analysis After that, the error rate comparison will change, as shown below.

From Table 3, it can be seen that the intelligent optimal algorithm of decision tree based on the analysis application model of research physical health test data and the comparison of error rate after use are reflected in the analysis index, comparison model, initial model, adjusted model, and error value. Among them, the analysis indicators are divided into modeling data and test data, and the comparison model is expressed as total error rate, high cost error rate, general cost error rate, and low cost error rate in the modeling data and test data. The total error rate, high cost error rate, and general cost error rate of modeling data show a decreasing trend in the overall value, and an increasing trend in the overall value of low cost error rate; the total error rate, high cost error rate, and general cost error rate of test data show a decreasing trend in the overall value, and an overall value of low cost error rate. There is an increasing trend. Therefore, the form of low cost error rate is negative in error value, which shows that there is no error in the test, and even the error control value is improved.

To sum up, the results of the actual calculation of the application mode of the analysis of physical health data by all the index elements substituted into the decision tree intelligent algorithm prove that the study of each index element of the analysis and processing system of physical health data by the decision tree intelligent algorithm has a certain significance for reference and presents a better benefit mode in the actual operation process and excellent feasibility.

## 5. Conclusion

With the continuous improvement of our basic living standards, the control and maintenance of the physical health of various groups in China has become one of the hot spots of public concern and gradually has become the main driving force to promote the development of medical industry in the actual operation process. Therefore, this paper takes the analysis and processing of physical health data as the research object, comprehensively discusses the analysis and processing mode of physical health data, analyzes the application of data analysis of physical health test and the intelligent algorithm model of decision tree, substitutes all index elements in the intelligent algorithm of decision tree, and summarizes that the intelligent algorithm of decision tree is based on the analysis of physical health test data, and through the example analysis to verify the feasibility of the algorithm, taking the student group in the university campus as the research object, it is concluded that there are numerical differences in the body mass index score, gender differences, and other elements of the physical health assessment mode, typical performance is that the control of modeling data and test data in each error rate is basically less than 15%, and in part of the research, the index shows negative value, which shows the effective control and adjustment ability of the algorithm for the error, and summarizes the analysis distribution diagram and the optimal algorithm mode of the decision tree intelligent algorithm model into the research school area. However, this paper only analyzes the impact of decision tree intelligent algorithm on the application of physical health test data from the university student group, lacking the research indicators and effects of other groups, so it will be improved in a more comprehensive research later.

## Figures and Tables

**Figure 1:** Use process of data management software of national youth group physical health standard.

**Figure 2:** Distribution of population sample analysis performed by the school algorithm.

**Figure 3:** Analysis of adolescent physical health test data under decision tree intelligent algorithm proportion of men and women.

**Table 1:** Data analysis and processing system of adolescent physical health.

System class	Specific indicators
User management	User account management
	User information management

Data upload	Physical examination score entry
	Introduction of physical test results

Data processing	Body measurement data increase
	Delete body measurement data
	Body measurement data modification
	Body measurement data query

Data standard management	Body measurement index management
	Scoring standard management

**Table 2:** Test data of adolescent body mass index after intelligent algorithm of decision tree.

Grade	Gender	Low weight range	Normal range	Overweight range	Obesity range
Freshman	Male	≤13.4	13.5–18.1	18.2–20.3	≥20.4
Sophomore	Male	≤13.6	13.7–18.4	18.5–20.4	≥20.5
Junior	Male	≤17.8	17.9–23.9	24–27.9	≥28
Senior	Female	≤17.1	17.2–23.9	24–27.9	≥28

**Table 3:** Intelligent optimal algorithm of decision tree based on research application model of health test data analysis and comparison of error rate after use.

Analysis index	Comparison model	Newly built model	Adjusted model	Error value
Modeling data	Total error rate (%)	8.42	8.29	0.13
	High cost error rate (%)	2.16	0.56	1.6
	General cost error rate (%)	12.25	10.75	1.5
	Low cost error rate (%)	12.88	15.69	−2.81

Test data	Total error rate (%)	9	8.17	0.83
	High cost error rate (%)	1.52	0	1.52
	General cost error rate (%)	10.99	9.4	1.59
	Low cost error rate (%)	17.82	17.95	−0.13

## Data Availability

The data used to support the findings of this study are included within the article.
